The article "Analysis of the Effects of Humidified High Flow Nasal Oxygen Therapy Combined with Noninvasive Mechanical Ventilation on Treatment Outcomes" was retracted in 2023. Reasons: signs of a paper mill; suspected computer-generated content; unreliable results or conclusions; lack of ethics approval or compliance.

# Analysis of the Effects of Humidified High Flow Nasal Oxygen Therapy Combined with Noninvasive Mechanical Ventilation on Treatment Outcomes

**DOI:** 10.1155/2022/2910813

**Published:** 2022-04-10

**Authors:** Hongjun Wang, Dawen Ma, Jingjing Hu, Qingxia Chu

**Affiliations:** ^1^Pulmonary and Critical Care Medicine, Pukou Branch, Jiangsu Province Hospital, Nanjing 211800, Jiangsu, China; ^2^Department of Physiology, Jiangsu Health Vocational College, Nanjing 211800, Jiangsu, China

## Abstract

**Objective:**

To investigate the effects of humidified high flow nasal cannula (HFNC) oxygen therapy combined with noninvasive mechanical ventilation (NIV) on blood gas indexes, complications, and respiratory function in patients with AECOPD.

**Method:**

100 patients with AECOPD admitted to the Department of Respiratory and Critical Medicine of Pukou District Central Hospital of Nanjing from March 2020 to February 2021 were selected. The patients were randomly divided into study group (50 cases) and control group (50 cases); both groups were given routine treatment such as bronchodilators, low-dose glucocorticoids, and antibiotics. During the treatment, the vital signs, inflammatory response indexes, fluid balance, and nutrition were continuously monitored; the body position was changed every 2 hours; and the curative effect was evaluated one week after treatment. On this basis, the control group received routine oxygen therapy combined with NIV (low flow conventional oxygen therapy + NIV), and the study group received HFNC combined with NIV (HFNC + NIV). The oxygen partial pressure (PaO2), peak expiratory flow rate (PEFR), arterial oxygen saturation (SaO2), first-second forced expiratory volume (FEV1), and mixed venous oxygen saturation (SvO2) level were compared between the two groups before and after treatment. Moreover, SECS scores before ventilation and 2, 4, 6, and 12 hours after ventilation were collected and analyzed. In addition, complications during oxygen therapy were compared.

**Result:**

Before treatment, there was no significant difference in the levels of PaCO2, FEV1, SaO2, PEFR, and SvO2 between the two groups (*P* > 0.05). After treatment, the levels of PaCO2 in the study group were lower than those in the control group, and the levels of FEV1, SaO2, PEFR, and SvO2 in the study group were higher than those in the control group *P* < 0.05(*P* < 0.05). There was no significant difference in SECS scores between the two groups before ventilation and 2 hours after ventilation (*P* > 0.05). The SECS scores of the study group at 4, 6, and 12 hours after ventilation were higher than those of the control group *P* < 0.05(*P* < 0.05). The total complication rate in the study group (8.00% vs. 24.00%) was lower than that in the control group (*P* < 0.05). Compared with low flow conventional oxygen therapy, NIV combined with HFNC can effectively reduce the incidence of complications in AECOPD patients during oxygen therapy, improve patients' ventilation comfort, and effectively improve blood gas indexes and respiratory function, with simple operation and high safety, which is worthy of clinical promotion and application.

The article "Analysis of the Effects of Humidified High Flow Nasal Oxygen Therapy Combined with Noninvasive Mechanical Ventilation on Treatment Outcomes" was retracted in 2023. Reasons: signs of a paper mill; suspected computer-generated content; unreliable results or conclusions; lack of ethics approval or compliance.

## 1. Introduction

Patients with mechanical ventilation will have various adverse conditions after tracheotomy, which will lead to hypoxemia. Therefore, oxygen therapy and nursing intervention should be strengthened to prevent hypoxemia. Chronic obstructive pulmonary disease (COPD) is a common disease characterized by persistent airflow limitation, which can be prevented and treated. The progressive development of airflow limitation is related to the enhancement of chronic inflammatory response of airway and lungs to toxic particles or gases. Acute exacerbation of chronic obstructive pulmonary disease (AECOPD) is dangerous and fatal. Its main clinical manifestation is respiratory dysfunction. In order to maintain normal respiratory function and stabilize vital signs, oxygen therapy is usually administrated to patients with AECOPD [1]. Compared to other oxygen administration methods, noninvasive mechanical ventilation (NIV) is easy to operate and inexpensive, so that it is currently the most widely used oxygen therapy for patients with AECOPD in clinical practice. However, insufficient facial compression, which happens in patients using NIV, can have negative impact on oxygen flow and on patients' eating and sleeping. Moreover, because the oxygen used in NIV is unheated dry cold gas, it is easy to cause sputum formation that reduces patients' comfortableness and tolerance during oxygen therapy [2]. In contrast, heated humidified high flow nasal cannula (HFNC) oxygen therapy, using high flow constant concentration humidified heated gas, can effectively improve patients' comfort and tolerance for continuous oxygen therapy. As a new oxygen therapy technology developed in recent years, HFNC has shown good clinical outcomes in patients with different respiratory diseases [3]. In this study, patients with AECOPD from the Central Hospital of Pukou District, Nanjing City, were selected as research participants to explore the effects of HFNC combined with NIV on blood gas parameters, complications, and respiratory function. The details are shown in the report.

## 2. Materials and Procedure

### 2.1. General Information

Using random number table method, a total of 100 patients with AECOPD who were admitted to the Department of Respiratory and Critical Care Medicine of Pukou District Central Hospital in Nanjing from March 2020 to February 2021 were divided into a study group (50 cases, receiving HFNC + NIV oxygen therapy) and a control group (50 cases, receiving low flow conventional oxygen therapy + NIV oxygen therapy). This study was approved by the Ethics Committee of Nanjing Pukou District Central Hospital. Inclusion criteria are as follows: (1) meeting the diagnostic criteria of AECOPD in “Guidelines for Diagnosis and Treatment of Chronic Obstructive Pulmonary Disease (2013 Revised Edition)” [4]; (2) partial pressure of carbon dioxide in the artery (PaCO2) ≥50 mmHg; (3) accepting the whole course of treatment in the hospital; (4) being conscious and able to breathe spontaneously; (5) being informed and willing to participate in the research. Exclusion criteria are as follows: (1) Acute Physiology and Chronic Health Evaluation-II (APACHE-II) [5] score ≥14; (2) comorbidities of other cardiovascular and respiratory diseases; (3) multiple organ failure; (4) fluid and electrolyte imbalance; (5) comorbidities of acute and chronic infection in other parts of the body; (6) comorbidities of mental/psychological disorders; (7) patients with hypoxemia before enrollment.

The article "Analysis of the Effects of Humidified High Flow Nasal Oxygen Therapy Combined with Noninvasive Mechanical Ventilation on Treatment Outcomes" was retracted in 2023. Reasons: signs of a paper mill; suspected computer-generated content; unreliable results or conclusions; lack of ethics approval or compliance.

The general data of the patients are as follows: the sex structure of the experimental group is 27 males and 23 females. The average age is 52.48 years, which is no more than 3.67 years. The sex structure of the control group was 26 males and 24 females. The average age is 51.95 years, which is no more than 3.85 years.

### 2.2. Treatment Procedure

#### 2.2.1. Oxygen Therapy

Both groups of patients were given conventional treatments such as bronchodilators, low-dose glucocorticoids, and antibacterial medications. During the treatment, vital signs, inflammatory response indicators, fluid balance, and nutrition were continuously monitored. Patient posture change was conducted every 2 hours while nurses assisted patients for sputum expectoration; intensive facial skin care was taken; and patients could communicate with the staff, drink fluid, and have meals. Treatment efficacy was evaluated one week later. Apart from these treatments, the control group received routine oxygen therapy combined with NIV therapy (low flow conventional oxygen therapy + NIV), which used a ventilator (Philips, DS700), pressure support ventilation + positive end-expiratory pressure mode, with an initial inspiratory pressure of 10 cmH2O, positive end-expiratory pressure of 4∼5 cmH2O, target tidal volume of 8∼10 ml/kg, and oxygen concentration of 30%–35%. The parameters were adjusted according to blood gas analysis results and eventually reached both PaCO2 <45 mmHg and partial pressure of oxygen (PaO2) > 60 mmHg. The study group received HFNC combined with NIV therapy (HFNC + NIV), which used a transnasal high flow humidified oxygen therapy system (Fisher & Paykel Company, RL-6000A) for high flow oxygen therapy via a warmed humidified nasal cannula with an initial flow rate of 40–50 L/min, oxygen concentration of 30%∼35%, and gas temperature of 37°C. The parameters were adjusted accordingly as blood gas analysis results changed, and finally reached both PaCO2 <45 mmHg and PaO2 >60 mmHg.

The article "Analysis of the Effects of Humidified High Flow Nasal Oxygen Therapy Combined with Noninvasive Mechanical Ventilation on Treatment Outcomes" was retracted in 2023. Reasons: signs of a paper mill; suspected computer-generated content; unreliable results or conclusions; lack of ethics approval or compliance.

#### 2.2.2. Nursing

All patients received routine nursing intervention during oxygen therapy: (1) Risk factor intervention. During oxygen therapy, risk factors such as airway infection, dust, hypertension, and hypercoagulability were closely monitored and controlled to prevent worsening airway inflammation that would affect patients' outcomes of oxygen therapy. (2) Respiratory care. During oxygen therapy, nurses on duty should detect airway complications based on patients' clinical information to improve the efficacy of oxygen therapy and prevent airway obstruction, and observe and evaluate patients' use of ventilator daily to avoid overuse of ventilator oxygen therapy and prevent patients from ventilator dependence. (3) Physical sign monitoring. Patients' respiratory rhythm, heart rate and rhythm, percutaneous oxygen saturation, central venous pressure, tidal volume, etc. were regularly monitored during oxygen therapy, and at the same time risk assessments were carried out to reduce the risk of mechanical ventilation complication. (4) Instrument and equipment care. During oxygen therapy, nurses on duty should pay attention to the patient's physical and mental state. If abnormal responses occur, symptomatic intervention should be carried out and the attending physician should be informed immediately. During oxygen therapy, disposable ventilator tubes should be used, and the pipe and ventilator humidifier should be regularly replaced to avoid lung infection caused by bacterial growth in the ventilator. (5) Psychological care. Patients were encouraged to actively communicate with family and friends to avoid prolonged isolation and development of negative psychological emotions, and at the same time patients' friends and relatives were warned not to display their own negative emotions that might affect the patient's mental state but to encourage the patient to actively participate in the treatment.

### 2.3. Observation Indicators

1. Comfort. The subjective comfort evaluation scale (SECS) [6] scores of the two groups before ventilation and at 2, 4, 6, and 12 hours after ventilation were collected and analyzed. The scale contains 10 scoring items with a total score of 100 points, and the score was directly proportional to the comfort level.
2. Blood gas parameters. Considering the patient's physical sign monitoring results, PaO2, SaO2, and mixed venous oxygen saturation (SvO2) levels before and after treatment were compared.
3. Respiratory function. Before and after treatment, forced expiratory volume in first second (FEV1) was measured by a pulmonary function instrument (SensorMedics, SQ7200) at the end of a forced inhalation, and peak expiratory flow rate (PEFR) was calculated through forced vital capacity curves.
4. Complications. Complications such as aspiration; dryness of the mouth, nose, and throat; nasal injury; and sputum expectoration disorders of the two groups were compared. The concurrent symptoms of patients were directly examined and compared by observation.

The article "Analysis of the Effects of Humidified High Flow Nasal Oxygen Therapy Combined with Noninvasive Mechanical Ventilation on Treatment Outcomes" was retracted in 2023. Reasons: signs of a paper mill; suspected computer-generated content; unreliable results or conclusions; lack of ethics approval or compliance.

### 2.4. Statistical Methods

SPSS software (version 22.0) was used for statistical analysis. *t*-tests were conducted for measurement data (age, PaCO2, body mass index, SaO2, APACHE-II, PaO2, SvO2, and SECS) that met normality and equal variances between groups, and *χ*^*2*^ tests were used for non-ordinal outcome categorical data (gender, satisfaction, and adverse events). *P* < 0.05 was considered statistically significant.

## 3. Results

### 3.1. Comparison of Baseline Data between the Two Groups

Comparing age (*t* = 0.775), body mass index (*t* = 0.037), PaCO2 (*t* = 0.422), APACHE-II score (*t* = 0.279), gender (*χ*^*2*^ = 0.069), and clinical classification (*Z* = 0.271) between the two groups, we found no statistically significant difference (*P* < 0.05) as shown in Table 1. SaO2 and SvO2 will be compared in the blood gas parameter. The age distribution statistics, the body mass index distribution, and the APACHE-II score at admission of the two groups of patients are illustrated in Figures 1–3, respectively.

### 3.2. Comparison of SECS Scores between the Two Groups at Each Time Point of Intervention

According to the traditional clinical medical standards, the SECS score is selected every two hours. In order to avoid the error of the experiment, the test is conducted again at 12 hours. There was no significant difference in SECS scores between the two groups before ventilation (*t* = 0.061) and 2 hours after ventilation (*t* = 0.922) (*P* > 0.05). However, the SECS scores of the study group were higher than those of the control group 4 hours (*t* = 2.865), 6 hours (*t* = 4.148), and 12 hours (*t* = 3.871) after ventilation. The differences were statistically significant (*P* < 0.05) as shown in Table 2. The SECS score line charts of the two groups of patients at each time point of intervention are shown in Figure 4.

The article "Analysis of the Effects of Humidified High Flow Nasal Oxygen Therapy Combined with Noninvasive Mechanical Ventilation on Treatment Outcomes" was retracted in 2023. Reasons: signs of a paper mill; suspected computer-generated content; unreliable results or conclusions; lack of ethics approval or compliance.

### 3.3. Comparison of Blood Gas Parameters between the Two Groups of Patients before and after Oxygen Therapy

PaO2 was selected to measure alveolar ventilation, SaO2 to measure oxygenation of lung and oxygen-carrying capacity of hemoglobin, and SvO2 to represent oxygen saturation of mixed venous blood. There was no significant difference in PaO2 (*t* = 0.042), SaO2 (*t* = 0.086), and SvO2 (*t* = 0.057) levels between the two groups before treatment (*P* > 0.05). The PaO2, SaO2, and SvO2 levels of the two groups after treatment were all higher than those of the same group before treatment; the PaO2 (*t* = 2.709), SaO2 (*t* = 2.538), and SvO2 (*t* = 3.139) levels for the study group were all higher than those of the control group after treatment; and the differences were statistically significant (*P* < 0.05) as shown in Table 3. The statistics of blood gas parameters before and after oxygen therapy for the two groups are illustrated in Figure 5.

### 3.4. Comparison of Respiratory Function between the Two Groups before and after Treatment

There was no significant difference in FEV1 (*t* = 0.120) and PEFR (*t* = 0.212) between the two groups before treatment (*P* > 0.05). Both the FEV1 and PEFR levels of the two groups after treatment were higher than those of the same group before treatment. After treatment, both FEV1 (*t* = 2.552) and PEFR (*t* = 2.314) of the study group were higher than those of the control group, and the difference was statistically significant (*P* < 0.05) as shown in Table 4.  Figure 6 shows the statistics of the respiratory function parameters of the two groups before and after treatment.

### 3.5. Comparison of Complications between the Two Groups

No severe complications such as airway spasms, absorption atelectasis, and oxygen toxicity occurred in either of the two groups during oxygen therapy. The total complication rate in the study group was lower than that in the control group (8.00% vs. 24.00%), and the difference was statistically significant (*χ*^*2*^ = 4.762, *P* < 0.05) as shown in Table 5.

## 4. Discussion

### 4.1. Severity of AECOPD

Chronic Obstructive Pulmonary Disease (COPD) has become a worldwide public health issue. Severity of COPD varies in different stages of the disease, among which AECOPD is dangerous and even fatal. AECOPD treatment should meet the long-term needs of patients, so as to achieve the goals of delaying disease progression, relieving symptoms, improving exercise tolerance, improving health status, preventing complications, preventing acute exacerbation, and reducing mortality. Patients mainly present with symptoms of persistent airway obstruction, such as coughing, breathing difficulty, wheezing, sputum expectoration, and pharyngeal discomfort. In addition, patients with AECOPD may suffer from respiratory failure due to upper airway obstruction and stenosis, which can severely affect their quality of life and health. Moreover, patients with AECOPD are prone to comorbidities or complications such as bronchial asthma (BA) and lower respiratory tract infection due to chronic mucosal injury. These conditions can cause continuous and recurrent damage to the respiratory system. Without active treatment, death may occur [7]. According to the data released by the World Health Organization, the fatality rate of AECOPD is as high as 11% for moderate to severe patients from routine admission and 20% for critically ill patients in the ICU. Respiratory complications are the major cause of death in AECOPD patients. Due to chronic airway inflammation, the risk of severe complications such as pulmonary heart disease, respiratory failure, and heart failure may increase, which subsequently elevates the risk of fatality [8]. Furthermore, the occurrence and development of AECOPD are closely related to environmental dust and toxic particles. With the aggravation of global industrial pollution problems, airway inflammation caused by airway harmful gases and particles exacerbates the symptoms (coughing, shortness of breath, fever, etc.) and vascular endothelial cell damage and increases the risk of airway obstruction, stenosis, and total occlusion, which greatly increases the mortality and disability rate of AECOPD patients and brings about serious challenges to public healthcare management nationally and globally.

The article "Analysis of the Effects of Humidified High Flow Nasal Oxygen Therapy Combined with Noninvasive Mechanical Ventilation on Treatment Outcomes" was retracted in 2023. Reasons: signs of a paper mill; suspected computer-generated content; unreliable results or conclusions; lack of ethics approval or compliance.

### 4.2. Pathogenesis of AECOPD

The pathogenesis of AECOPD has not yet been fully understood. However, clinical studies suggest that chronic inflammation in the airways and lungs and neutrophil aggregation induced by allergic immune responses are the main causes of AECOPD. For example, Cao et al. [9] suggested that the release of histamine triggered by the stimulation of toxic gases and particulate matter in the respiratory system is the main influencing mechanism of AECOPD allergic immune response inflammation. Normally, the blood level of immunoglobulin *E* in humans is low. However, when the airway and lungs are stimulated by allergens such as pollen, dust, toxic gases, chemicals, and cigarettes, allergic immune responses occur in the body, which elevates serum IgE levels and aggravates damage to the airway and lungs resulting in chronic noninfectious inflammation. Yang et al. [10] pointed out that IgE antibodies in the human body are mainly secreted by plasma cells produced by B lymphocytes under the stimulation of antigens. Usually, this process is a normal defense regulation mechanism of the organism, which is beneficial for the body to protect itself from exogenous pathogen invasion and increase the body's ability of resistance. Nevertheless, due to physical condition and chronic respiratory diseases, people who are suffering from AECOPD have an abnormally high levels of serum and respiratory mucosal immunoglobulin *E* under the stimulation of airway toxic particles and chemical substances, leading to unusual release of IgE-mediated histamine. This can further induce abnormal secretion of neutrophil elastase and neutrophil aggregation leading to allergic immune responses of the airway and lungs, with functional impairment, and also causing abnormal mucus secretion that blocks the airway.

The article "Analysis of the Effects of Humidified High Flow Nasal Oxygen Therapy Combined with Noninvasive Mechanical Ventilation on Treatment Outcomes" was retracted in 2023. Reasons: signs of a paper mill; suspected computer-generated content; unreliable results or conclusions; lack of ethics approval or compliance.

### 4.3. Current Treatment for AECOPD

Clinical treatment for patients with AECOPD aims to reduce the risk of death and minimize damage to the respiratory system through alleviating airway inflammation, improving airway gas flow, and relieving airway symptoms. Commonly used medications in clinical treatment for AECOPD include glucocorticoids (GCs), antibiotics, bronchodilators, and leukotriene receptor antagonists [11]. Patients should be informed that antibiotics must be used under the guidance of doctors; antibiotics should not be used for a long time, usually 7 days to 14 days, to avoid dysbacteriosis; for oral administration, plenty of water should be drunk after taking sulfanilamide drugs to avoid crystallization of urine, and less water should be drunk after taking cough syrup to avoid affecting the curative effect. Exacerbation of COPD is often caused by respiratory system infection, of which common susceptible pathogens for AECOPD include *Mycoplasma pneumoniae*, *Haemophilus influenzae*, *Streptococcus pneumoniae*, *Moraxella catarrhalis*, and viruses. Therefore, antibacterial agents are very important in treating AECOPD [12]. Selecting antibiotics is mainly based on the results of bacterial culture. For patients who have positive sputum culture results, antibacterial drugs should be selected according to the pathogenic strains of the infection. For patients with mild symptoms of infection, it is suggested that they do not use antibiotics at all, or use standard (non-broad-spectrum) antibiotics, for example, choosing penicillin for Gram-positive bacteria, to avoid pathogen resistance caused by antibiotics overuse. For patients with moderate to severe infection, it is recommended that they use broad-spectrum antibiotics, such as piperacillin-tazobactam, levofloxacin, and ceftriaxone, as early as possible to control infection progression, and the antibiotics should be adjusted according to the results of the sputum culture and drug sensitivity test [13]. In addition, glucocorticoids are steroid hormone medicines with good immune regulation and anti-inflammatory effects. They can rapidly relieve the airway and lung inflammatory symptoms and pathological immune response, thereby reducing immune dysfunction and respiratory system inflammation damage and easing clinical symptoms of AECOPD. Currently, there are two main administration routes for glucocorticoids: oral administration and inhalation. Oral administration, predominantly including hydrocortisone, prednisone, and dexamethasone, is convenient and has little restrictions on patients' physical and pathological conditions. However, because oral formulation reaches the whole body systemically instead of accurately targeting respiratory tract lesions, both its effective time and clinical efficacy are inferior to those of inhaled formulation [14]. Moreover, aerosol inhalation can directly deliver medicine to respiratory tract lesions, which is convenient and quick, requires small dosages, has few side effects, and is easily accepted by the patient. At present, using inhaled GCs is still the first line treatment for AECOPD recommended by major guidelines. With the continuous advancing of clinical pharmaceutical technology, inhaled GCs as finer particles are gradually being applied to the treatment of AECOPD. While traditional GCs aerosol particles for inhalation usually reached 2.0∼4.0 *μ*m in the past, the diameter of aerosol particles of modified GCs is less than 2.0 *μ*m, of which aerosol particles can enter small airways. Finer particle inhalation produces better outcomes with relatively even particle deposition and distribution [15]. As persistent airflow obstruction is the main symptom of AECOPD, bronchodilators are also basically used to treat AECOPD, among which *β*2 receptor agonist (terbutaline, salbutamol, salmeterol, etc.) bronchodilators can selectively affect airway smooth muscle receptors, thereby inhibiting bronchoconstriction, improving the efficiency of airway gas passage, and enhancing respiratory function [20]. Nevertheless, anticholinergic (tiotropium bromide, ipratropium bromide, etc.) bronchodilators can effectively dissolve airway secretion, lubricate respiratory tract, and expand the bronchus, thereby promoting the secretion of lung surfactant substances and ciliary movement, dredging airway, and reducing mucosal irritation in the respiratory tract, resulting in better outcomes of airflow in patients with AECOPD [16].

The article "Analysis of the Effects of Humidified High Flow Nasal Oxygen Therapy Combined with Noninvasive Mechanical Ventilation on Treatment Outcomes" was retracted in 2023. Reasons: signs of a paper mill; suspected computer-generated content; unreliable results or conclusions; lack of ethics approval or compliance.

### 4.4. The Importance of Oxygen Therapy in the Treatment of AECOPD

Pharmaceutical treatment can effectively control the progress of AECOPD, and after systemic treatment, clinical symptoms can be relieved, and most patients gradually transit to a stable phase. However, due to slow therapeutic effect and rapid onset of AECOPD, apart from route medicine administration to control the condition, oxygen therapy and artificial ventilation are also required to maintain respiratory function and stabilize vital signs. Therefore, in addition to conventional pharmaceutical treatment, oxygen therapy is also important to eliminate clinical symptoms and improve prognosis quality in patients with AECOPD [17, 18]. In clinical practice, oxygen therapy is often used to assist AECOPD patients for normal gas exchange and maintain stable vital signs, but different ventilation modes vary in comfortableness, tolerance, and effectiveness [19–21]. The oxygen flow rate is continuous and low, the oxygen concentration is generally 24% ∼ 30%, and the flow rate is 1 l/min ∼ 2 l/min. Inhaled oxygen must be humidified to avoid dryness of nasal mucosa and discomfort. NIV is widely used in clinical oxygen therapy for patients with AECOPD due to its economical advantage and convenience. However, it has disadvantages such as strong irritation of dry and cold gas, flow instability, and strong discomfort. Patients tend to have low tolerance due to dry and cold gas irritating the respiratory tract, and high reintubation rate after the extubation. This may prolong oxygen therapy time and increase comprehensive treatment cost, which has certain limitations [22–24]. With the continuous development of clinical oxygen therapy technology, HFNC is gradually used for patients with AECOPD. This technology can simulate the physical state of normal inhaled gas in the human respiratory tract by heating and humidifying the therapy oxygen, which can effectively improve patients' comfort and tolerance during oxygen therapy, and reduce dry and cold air irritation in the respiratory tract so as the impact on patients' recovery [25].

### 4.5. Analysis of Research Results

This study explored the effects of HFNC combined with NIV on blood gas parameters, complications, and respiratory function in patients with AECOPD. Our study results showed that PaO2, SaO2, and SvO2 levels of the study group after treatment were higher than those of the control group, and SECS scores at 4, 6, and 12 hours after ventilation were higher than those of the control group. This is largely consistent with the study by Chen and Liu [21], indicating that compared to conventional NIV, HFNC combined with NIV has a higher degree of comfort, can increase patient compliance in oxygen therapy, and can improve blood gas parameters. The results also showed that FEV1 and PEFR levels of the study group after treatment were higher than those of the control group, and the total complication rate (8.00% vs. 24.00%) during treatment period was lower than that of the control group. This is in line with the study by Tan et al. [24], indicating that HFNC combined with NIV can further improve respiratory function in patients with AECOPD and reduce the risk of complications. On analyzing the reasons for the differences in the above results, it was suggested that HFNC oxygen therapy improves gas biocompatibility through the process of heating and humidification, which reduces low temperature dry gas irritation to the respiratory tract, further improves blood gas parameters and respiratory function, and decreases incidence rate of complications. Moreover, compared to using NIV alone, the addition of HFNC can increase gas flow and flow stability and improve patients' comfort. It is worth noting that due to the restrictions of funding, personnel, time, and other factors, this study has limitations such as the small sample size, short observation period, and few observation indicators, which may lead to study result deviations from clinical practice. Nevertheless, it has provided some empirical evidence value for further research.

The article "Analysis of the Effects of Humidified High Flow Nasal Oxygen Therapy Combined with Noninvasive Mechanical Ventilation on Treatment Outcomes" was retracted in 2023. Reasons: signs of a paper mill; suspected computer-generated content; unreliable results or conclusions; lack of ethics approval or compliance.

## 5. Summary

In summary, the combination of NIV and HFNC can effectively reduce incidence rate of complications in AECOPD patients during oxygen therapy, increase ventilation comfort, and improve blood gas indicators and respiratory function. This oxygen therapy regimen is simple to operate and economical and does not have high staffing and equipment requirements, which is suitable for most clinical hospitals. It can bring about positive changes in the quality of hospital care services and is worthy of clinical promotion and application.

## Figures and Tables

**Figure 1:** Statistical chart of patients' age distribution in the two groups.

**Figure 2:** Statistical chart of patient body mass index distribution in the two groups.

**Figure 3:** Statistical chart of APACHE-II score distribution of the two groups of patients.

**Figure 4:** SECS score line chart of two groups of patients at each time point of intervention.

**Figure 5:** Statistical chart of blood gas indexes of the two groups of patients before and after oxygen therapy.

**Figure 6:** Statistical chart of respiratory function indexes of the two groups before and after treatment.

**Table 1:** Comparison of baseline data between the two groups of patients.

Group	*n*	Age (years)	BIM (kg/m^2^)	PaCO2 (mmHg)	APACHE-II (min)	Gender		Disease classification			
						Male	Female	Grade I	Grade II	Grade III	Grade IV
Research group	50	52.48 ± 3.67	24.62 ± 4.34	57.43 ± 2.12	10.59 ± 2.13	27 (54.00)	23 (46.00)	0 (0.00)	0 (0.00)	41 (82.00)	9 (18.00)
Control group	50	51.95 ± 3.85	24.59 ± 4.53	57.35 ± 2.20	10.48 ± 2.20	26 (52.00)	24 (48.00)	0 (0.00)	0 (0.00)	43 (86.00)	7 (14.00)
*χ* ^2^ */t*		0.775	0.037	0.422	0.279	0.069		0.271			
*P*		0.440	0.970	0.537	0.780	0.792		0.965			

The article "Analysis of the Effects of Humidified High Flow Nasal Oxygen Therapy Combined with Noninvasive Mechanical Ventilation on Treatment Outcomes" was retracted in 2023. Reasons: signs of a paper mill; suspected computer-generated content; unreliable results or conclusions; lack of ethics approval or compliance.

**Table 2:** Comparison of SECS scores between the two groups at each time point of intervention (*x* ± *s*).

Group	*n*	Before ventilation	Ventilation for 2 hours	Ventilation for 4 hours	Ventilation for 6 hours	Ventilation for 12 hours
Research group	50	78.52 ± 7.63	62.13 ± 5.58	66.56 ± 5.28	70.15 ± 4.29	72.13 ± 5.57
Control group	50	78.43 ± 7.24	61.13 ± 5.26	63.56 ± 5.19	66.46 ± 4.60	68.20 ± 4.53
*t*		0.061	0.922	2.865	4.148	3.871
*P*		0.952	0.359	0.005	<0.001	<0.001

**Table 3:** Comparison of blood gas indexes between the two groups before and after treatment (*x* ± *s*).

Group	*n*	PaO2 (%)		SaO2 (%)		SvO2	
		Before treatment	After treatment	Before treatment	After treatment	Before treatment	After treatment
Research group	50	6.70 ± 2.13	14.62 ± 3.11^*∗*^	70.62 ± 4.79	98.89 ± 7.26^*∗*^	54.35 ± 6.11	75.19 ± 8.95^*∗*^
Control group	50	6.65 ± 2.08	10.53 ± 2.95^*∗*^	71.06 ± 5.13	89.59 ± 8.13^*∗*^	54.52 ± 6.23	68.76 ± 7.84^*∗*^
*t*		0.042	2.709	0.086	2.538	0.057	3.139
*P*		0.967	0.000	0.904	0.000	0.946	0.000

Note. Compared with before treatment in this group, ^*∗*^*P* < 0.05.

**Table 4:** Comparison of respiratory function between the two groups before and after treatment (*x* ± *s*).

Group	*n*	FEV1 (L)		PEFR (L/s)	
		Before treatment	After treatment	Before treatment	After treatment
Research group	50	2.03 ± 0.79	2.63 ± 0.65^*∗*^	3.26 ± 0.89	3.95 ± 0.76^*∗*^
Control group	50	2.05 ± 0.80	2.29 ± 0.62^*∗*^	3.22 ± 0.91	3.60 ± 0.68^*∗*^
*t*		0.120	2.552	0.212	2.314
*P*		0.905	0.012	0.833	0.023

Note. Compared with before treatment in this group, ^*∗*^*P* < 0.05.

**Table 5:** Comparison of incidence of complications between the two groups [*n* (%)].

Group	*n*	Obstruction of expectoration	Aspiration	Nasal injury	Dry mouth and nasopharynx	Total adverse events
Research group	50	2 (4.00)	1 (2.00)	1 (2.00)	0 (0.00)	4 (8.00)
Control group	50	4 (8.00)	2 (4.00)	3 (6.00)	3 (6.00)	12 (24.00)
*χ* ^*2*^						4.762
*P*						0.029

## Data Availability

No data were used to support this study.
